This article has been retracted.

# Imaging Diagnosis of Primary Solitary Bone Neoplasts and Its Comparison with Tumor-like Lesions

**DOI:** 10.1155/2022/2692539

**Published:** 2022-08-12

**Authors:** Xuying Wei, Wenxin Zheng, Wencai Tang

**Affiliations:** Radiology Department, The Second Affiliated Hospital of Hainan Medical University, Haikou, Hainan, China

## Abstract

**Objective:**

To explore the imaging diagnostic value of primary solitary bone tumor and tumor-like lesion of iliac crest.

**Methods:**

A total of 156 patients with primary solitary bone tumors and tumor-like lesions of the iliac bone treated in our hospital were selected, and the patients were diagnosed by X-ray, CT, and MRI. Sexual analysis of single diagnostic and combined diagnostic value was carried out.

**Results:**

Round high-density shadow, soft tissue mass shadow, soft tissue mass, right intestinal tube, and bladder obvious pressure were observed. The detection rates of giant cell tumor of bone, myeloma, osteochondroma, chondroma, eosinophilic granuloma, osteosarcoma, fibrous dysplasia, and Hodgkin lymphoma were 34.6%, 12.8%, 11.5%, 10.3%, 7.7%, 6.4%, 3.8%, and 2.6%, and the differences were statistically significant (P < 005); X-ray, CT, MR single diagnostic comparison, three methods joint diagnostic missed diagnosis rate and misdiagnosis rate, higher detection rate (*P* < 0.05); combined with X-ray, CT, MR single diagnosis, three methods joint diagnosis sensitivity, specificity, accuracy, statistical significance (*P* < 0.05); comparison with X-ray, CT, MR single diagnosis, three methods jointly diagnosed *positive* predictive value, negative predictive value higher, difference statistics significance (*P* < 0.05); there is a significant difference in the near-end, backbone, and distal detection rate of different bone tumors and tumor lesions, including the humerus and tibia. There is a statistical significance of the detection rate, and the difference is*P* < 0.05.

**Conclusion:**

X-ray plays an important role in the diagnosis of primary solitary bone tumor and tumor-like lesion of iliac crest and is the first choice in clinical diagnosis. In the diagnosis of tumor disease, range, and soft tissue mass, MRI and CT diagnostic value can provide effective theoretical basis for patient clinical treatment. Therefore, the appropriate diagnostic method should be selected according to the specific situation of the patient, so that the efficiency of the clinical feature is improved.

## 1. Introduction

Data statistical results showed the crowd of cartilantic tumors in the middle of the 40-year-old population changes with age, and the chance of chondrosarcoma will also change [1]. Primary malignant bone tumors mainly occur in long bones of the limbs, which increases the difficulty of imaging diagnosis due to various types of tumors [2]. Iliac bone lesions are more common, such as flat bones with abundant red bone marrow, and myeloma and metastatic tumors are also more common. Metastatic tumors account for about 31% of pelvic tumors. However, single tumor-like lesions and primary tumors of the iliac bone are not common, and eosinophilic granuloma and chondroma are common [3, 4].

There are relatively many clinical reports on Ewing tumor, metastatic tumor, myeloma, and non-Hodgkin lymphoma, but there are few reports on primary solitary bone tumor and tumor-like lesions of the iliac crest [5]. Primary solitary bone tumors and tumor-like lesions of the iliac bone greatly interfere with the normal life of patients. Therefore, it is necessary to accurately diagnose patients and formulate treatment plans based on imaging features. In this study, 156 patients with primary solitary bone tumors and tumor-like lesions of the iliac bone treated in our hospital were selected as the research objects, which are representative of the research objects. The patients were diagnosed by X-ray, CT, and MRI, respectively. Imaging features of primary solitary bone tumors and tumor-like lesions, to explore the detection rates of different types of bone tumors and tumor-like lesions in the proximal, diaphysis, and distal ends and to evaluate the dynamic changes of primary solitary bone tumors and tumor-like lesions of the iliac bone situation, discover its changing laws and causes and provide a basis for the treatment of the disease. The relevant content is now reported as follows.

## 2. Data and Methods

### 2.1. General Information

A total of 62 patients with primary isolated bone tumor and tumor-like lesion of iliac crest treated in our hospital were selected for X-ray. All subjects included in this study did not drop out. CT and MRI diagnosis were performed successively. There were 62 patients, including 37 males and 25 females, with an average age of 46.0 ± 19.2 years, an average body weight of 56.8 ± 8.7 kg, and an average BMI of 21.0 ± 2.2 kg/㎡. The subjects agreed to this study, which was approved by the hospital ethics committee.

### 2.2. Inclusion Criteria

The inclusion criteria were as follows: (1) According to the “Guidelines for Clinical Evidence-Based Diagnosis and Treatment of Osteosarcoma” [6], patients were diagnosed with primary solitary bone tumor and tumor-like lesions of the iliac bone. (2) The initial site of tumor is the bone. (3) Patients with multifocal or single-focal lesions diagnosed by imaging were included. (4) Patients with normal cognitive function can cooperate with the study.

### 2.3. Exclusion Criteria

The exclusion criteria were as follows: (1) patients with autoimmune diseases; (2) patients who were not followed up for clinical prognosis; (3) patients during pregnancy or lactation; (4) patients with mental illness.

### 2.4. Termination Criteria

The termination criteria were as follows: (1) patients who do not comply with the approved protocols or relevant regulations; (2) patients with sudden adverse events; (3) patients lost to follow-up; (4) patients who voluntarily withdraw their informed consent.

## 3. Method

The X-ray machine (GeRevolutionxR/*D*) is used for the X-ray diagnosis of the frontal pelvis. CT diagnosis included the following scanning parameters: the slice thickness, 5–10 mm; matrix, 512 × 512; voltage, 100–120 kV; current, 140–200 mAs; and reconstruction interval, 1.0–1.25 mm. 3.0 T superconductive MR core magnetic resonance unit was applied to perform MR-enhanced scan for patients, using 70–90 ml omnipac via cubital vein mass injection.

### 3.1. Observation Indicators

#### 3.1.1. Patient Baseline Data Analysis

Baseline data included gender, age, weight, BMI, and other materials.

#### 3.1.2. Imaging Features of Primary Isolated Bone Tumors and Tumorigenic Lesions of Iliac Crest

Conditions such as metastasis, myeloma, osteochondroma, chondroma, eosinophilic granuloma, Ewing sarcoma, osteosarcoma, fibrodysplasia, and Hodgkin's lymphoma were measured, and the detection rate was calculated.

#### 3.1.3. Diagnostic Value of Primary Isolated Bone Tumor and Tumor-like Lesion-Type Metastases of the Ilium

It was predicted using diagnostic rate, missed diagnosis rate, misdiagnosis rate, sensitivity, specificity, accuracy, positive predictive value, and negative predictive value.

#### 3.1.4. Comparison of the Detection Rates of Different Types of Bone Tumors and Tumor-like Lesions

The cases of an examination on the humerus, tibia, proximal fibula, ulna, radius, and femur are counted.

### 3.2. Statistical Method

The collected data were input into EXCEL, and the statistical software SPSS22.0 was used for data analysis. The normal distribution test was carried out using the collected data. If the data met the normal distribution, the composition ratio and rate were used to describe the counting data, and the Chi-square test was used to analyze the difference between groups. The *T* test was used to analyze the difference between groups. Logistic regression was used to analyze the influencing factors of physical fitness in the case group, and *P* < 0.05 was considered to be statistically significant. GraphPadPrism8 was used in the study.

## 4. Results

### 4.1. Analysis of the Baseline Data in 156 Patients

The study included 82 males and 74 females, with an average age of 46.0 ± 19.2 years, an average body weight of 56.8 ± 8.7 kg, and an average BMI of 21.0 ± 2.2 kg/m^2^ (Table 1).

### 4.2. Imaging Features of Primary Isolated Bone Tumors and Tumor-like Lesions of the Iliac Crest

Features such as round high-density shadow, soft tissue mass shadow, soft tissue mass, and obvious compression of the right intestine and bladder were observed (Table 2).

### 4.3. Primary Solitary Bone Tumor and Tumor-like Lesion-Type Metastases of the Iliac Crest

The detection rates of metastasis, myeloma, osteochondroma, chondroma, fibrodysplasia, Ewing sarcoma, eosinophilic granuloma, osteosarcoma, and Hodgkin's lymphoma were 30.6%, 14.5%, 12.9%, 1.6%, 4.8%, 4.8%, 1.6%, 1.6%, and 1.6% (Figure 1).

By contrast, in diagnostic methods of X-ray, CT, and MR, the diagnostic values were statistically significant (*P* < 0.05) (Figure 2).

By contrast, in diagnostic methods of X-ray, CT, and MR, the diagnostic values were statistically significant (*P* < 0.05) (Figure 3).

By contrast, in diagnostic methods of X-ray, CT, and MR, the diagnostic values were statistically significant (*P* < 0.05) (Figure 4).

Near-end, backbone, and distal detection rates of different bone tumors and distal detection rates, have significant differences in the near-end, backbone and distal detection rate of different bone tumors and tumor morphology, including humerus, tibia, tibia proximal And the blem, the distal radius, and the femoral femur is relatively high, and the detection rate comparisons, the difference is statistically significant (*P* < 0.05) (Figure 5).

## 5. Discussion

At present, the etiology of bone tumors is not very clear, but the occurrence of bone tumors is an extremely complex process, which is the result of the combined effects of genetic factors, environmental abnormalities, and toxic exposure. Genetics is the most important factor. If there is a family history of malignant bone tumor, the incidence rate is higher than that of the general population. Bone pain, arthralgia, and movement disorders are considered bone tumors; however, many bone tumors do not have typical clinical symptoms in the early stage, so it is difficult to detect early. Bone tumors are usually benign in the initial stages of the disease, but as the disease progresses, they can develop around the bone and even compress the surrounding soft tissue cells, causing pain. When this pain occurs, it means that the disease has progressed to the middle and late stages. Bone tumor formation is a very complex process, with many different genetic changes affecting different transmission pathways. Variations in some genes can lead to similar functional outcomes and produce similar tumors. All tumors have many changes in transmission pathways at the same time. Genetic mutations may have indirect or secondary effects, with tumors overexpressing normal growth factors or receptors, cytokines, and enzymes, allowing tumor cells to invade tissues, recruit new blood vessels, and even form distant metastases. These molecular biological processes are not associated with mutated genes but can be used as new biotherapeutic targets. According to the different nature of primary bone tumor, it is divided into benign bone tumor and malignant bone tumor. After the diagnosis of primary bone tumor, surgery is usually the first choice to remove the tumor.

The tibia has an irregular characteristic, which is the body's maximum flat bone, which is a large number of bone tumors, with the proportion of metastasis than being relatively high, and other bone marrow tumors, bone malignant lymphoma [7–9]. Clinical data show that the incidence of ilibular disease in the primary malignant bone tumor is about 9.6%, of which the patient is high in chondrosatoma is high, and it is an osteosarcoma, and Juventi meat [10–12]. This study analyzed primary solitary bone tumors and tumor-like lesion-type metastases of the iliac bone, including giant cell tumor of bone, myeloma, osteochondroma, chondroma, eosinophilic granuloma, osteosarcoma, osteosarcoma, fibrous dysplasia, and Hodgkin's lymphoma. The detection rates were 34.6%, 12.8%, 11.5%, 10.3%, 7.7%, 6.4%, 6.4%, 3.8%, 3.8%, and 2.6%. The results of this study are consistent with those of other clinical scholars, and the results are credible and have high promotion value and significance. The results confirmed that giant cell tumor of bone, myeloma, and osteochondroma were the primary solitary bone tumors of the iliac bone and the main metastatic tumors of tumor-like lesions.

Osteopolysis is obvious in tumor-like lesions, and the characteristics of iliac tumor lesions are obvious. Most tumor patients will have soft tissue mass that plays an important role in the clinical diagnosis of skeletal lesion [13]. The discrepancy is no statistically significant [14]y[15]. The bone cortex thickening or thinning is the main imaging characteristics of chondrosarcoma. It often has a soft tissue mass, and the main form of the lesion is a circular arc shape, with internal flute calcification, spot shape or annular, and there is a difference in calcification of different soft bone tumors [16]. The study analyzed the image characteristics of primary isolated bone tumor and tumor morphology of the iliac bone, and the results showed that the round high-density shadow, soft tissue swelling, soft tissue mass, right bowel, and bladder were significantly compressed [17]. The results confirmed that there is a lesionic imaging characteristics to identify a variable and malignant tumor, often through the osteospondel cartilage cap, osteogenic protrusion, soft tissue mass, tumor calcification, plaque shape, jet tumor bone, and clinical diagnosis, which can be used for diagnosis and formulation of treatment options [18]. It is worth noting in clinical diagnosis, which should be distinguished from the bone and hardened myelitis. The tuberculous joint surface is easily destroyed, where the ankle joint is the main part, and it can easily cause cold abscess [19].

The clinical common diagnostic method of iliac crest tumor morbidity is *X*-ray extensive diagnosis, which can show most of the bone damage, especially in the diagnosis rate of overlapping diagnosis of the iliac crest [20]. However, due to the more of the bone structure, the structure is complex, the common intestinal content, intestinal gas and other factors, pelvic soft tissue, mild bone damage and soft tissue mass, missed diagnosis and misdiagnosis, and this will affect the diagnosis accuracy [21]. Therefore, the diagnostic method can improve the diagnostic accuracy and ensure good photographing conditions, which requires cleaning of the intestines. If the iliac lesion has a change in soft tissue, this will affect the X-ray diagnosis, so it is necessary to add MRI and CT diagnostics [22]. At present, imaging technology has continuously developed, and the image is not clearly displayed by CT diagnosis, which can be made up of the flat film, and the clinical diagnosis rate is significantly improved [23]. The CT diagnostic advantage of the iliac bone tumor and tumor-like lesions is obvious. Firstly, it is possible to clarify the internal structure and mass of the tissue and determine the calcification of tissue mass and show the degree of enhancement [24]. Secondly, it can be display the soft tissue mass and the surrounding tissue relationship. Thirdly, the X-ray diagnostic defect makes up for the bone reaction. Fourthly, CT diagnosis can be multiorientation, multiplane display lesion, size, and morphology, while showing the interval anatomical relationship and osteoporous change range [18]. Currently, in the diagnosis of the primary isolated bone tumors and tumor morbidity, CT and MRI diagnoses are increasingly widely used, can more accurately judge the osteoporous variation, and will show the tibia failure. They can timely evaluate whether the iliac bone signal is abnormal, which provides a good basis for the diagnosis of disease [25]. More and more academic researchers pay attention to the imaging diagnosis of primary solitary bone tumors and tumor-like lesions of the iliac bone. X-ray and CT are used to diagnose patients. Two of the 20 patients have the “floating ice sign,” the boundary is blurred, there will be residual bone density sclerosis and increase, and the original bone shape and contour are still maintained. Studies confirmed this conclusion. This study analyzed the diagnostic value of X-ray, CT, and MRI in bone tumors and tumor-like lesions. The results showed that the diagnostic rates of X-ray, CT, MRI, and combined diagnosis were 5.8%, 3.2%, 1.3%, and 0.6%, respectively, and the missed diagnosis rates were 4.5%, 1.9%, 0.0%, and 0.0%, respectively. The misdiagnosis rates were 89.7%, 94.9%, 98.7%, and 99.4%, respectively. Compared with X-ray, CT, and MRI single diagnosis, the combined diagnosis rate of the three methods was higher, the rate of missed diagnosis and misdiagnosis was lower, and the rate of missed diagnosis and misdiagnosis was lower. The detection rate, sensitivity, specificity, and accuracy were higher than those of other diagnostic methods, and the differences were statistically significant (*P* < 0.05). Different diagnostic methods have different characteristics and advantages. The clinical should choose the appropriate diagnosis method according to the age, the onset site, soft tissue mass, and osteopoly damage imaging characteristics. If there are difficulties in diagnosis, it should be combined with pathological diagnosis. The study explores the proximal end, backbone, and distal end detection rate of different bone tumors and tumor lesions. The results show that there is a significant difference in the near-end, backbone, and distal end detection rate of different bone tumors and tumor diseases, and there were statistical discrepancies in the diagnosis of humerus, tibia, distal radius, and femur (*P* < 0.05). The results of the study were consistent with the study results of clinicians, and the clinical reference value was higher [26].

This study can analyze the detection rates of the proximal end, backbone, and distal end of different bone tumors and tumor-like lesions in order to find out the disease progression. The structure of the paper is designed reasonably. However, there are still deficiencies that need to be improved. The study only analyzed the difference between single diagnosis and combined diagnosis of X-ray, CT, and MRI and did not analyze the combination of the two detection methods. This problem needs to be investigated in the research. Further lucubrate is needed to improve the accuracy of the study.

## 6. Conclusion

X-ray plays an important role in the clinical diagnosis of primary solitary bone tumors and tumor-like lesions of the iliac crest and is the preferred diagnostic method. MRI and CT have higher diagnostic value in tumor lesion staging, scope, and soft tissue mass diagnosis, which can provide effective theoretical basis for clinical treatment of patients. Therefore, the appropriate diagnostic method should be selected according to the specific situation of the patient, and the efficiency of the clinical feature shall be improved.

## Figures and Tables

**Figure 1:** Primary solitary bone tumor and tumor-like lesion-type metastases of the iliac crest.

**Figure 2:** X-ray, CT, and MRI diagnosis: missed diagnosis rate and misdiagnosis rate.

**Figure 3:** Diagnostic value of X-ray, CT, and MRI.

**Figure 4:** X-ray, CT, and MRI diagnosis: positive predictive value and negative predictive value.

**Figure 5:** Proximal, diaphyseal, and distal detection rates of different bone tumors and tumor morphologies.

**Table 1:** Analysis of patient baseline data.

General clinical data		
Gender	Male	37
	Female	25
Average age (years)		46.0 ± 19.2
Average weight (kg)		56.8 ± 8.7
Average BMI (kg/m^2^)		21.0 ± 2.2

**Table 2:** Imaging features of iliac crest isolated osteotic neutral tumors and tumor morphology (*N* (%)).

Imaging characteristics	Count	Proportion (%)
Uniform length T1, long T2 signal	10	6.4
Soft tissue swellings in the disease	20	12.8
Soft tissue mass	18	11.5
The bone expansion is thin, the elliptical changes, the hardening edge is surrounded, and the boundary is clear	6	3.8
Point-to-spot calcification	12	7.7
Ankle joint, gap blur, soft tissue mass	10	6.4
Interpretation of irregular calcification in tissue mass, no bone film reaction	6	3.8
High-tertiary, multicircular, high density	54	34.6
T1WI medium signal and T2WI high signal disease in the iliac crestand tibia, and the bone marrow cavity in the lesion can be reinforced	4	2.6
Right bowel and bladder are obviously compressed	16	10.3

## Data Availability

All data generated or analyzed during this study are included in this article.
